The article "Imaging Manifestations and Evaluation of Postoperative Complications of Bone and Joint Infections under Deep Learning" was retracted in 2023. Reasons: signs of a paper mill; compromised peer review; unreliable results or conclusions.

# Imaging Manifestations and Evaluation of Postoperative Complications of Bone and Joint Infections under Deep Learning

**DOI:** 10.1155/2021/6112671

**Published:** 2021-12-20

**Authors:** Wei Mao, Xiantao Chen, Fengyuan Man

**Affiliations:** ^1^Department of Orthopedics, Capital Medical University, Beijing 100000, China; ^2^Department of Osteonecrosis of the Femoral Head Luoyang Orthopedic Hospital of Henan Province, Orthopedics Hospital of Henan Province, Luoyang 471000, China; ^3^Department of Radiology, Capital Medical University, Beijing 100000, China

## Abstract

To explore and evaluate the imaging manifestations of postoperative complications of bone and joint infections based on deep learning, a retrospective study was performed on 40 patients with bone and joint infections in the Department of Orthopedics of Orthopedics Hospital of Henan Province of Luoyang City. Sensitivity and Dice similarity coefficient (DSC) were used to evaluate the image results by convolutional neural network (CNN) algorithm. Imaging features of postoperative complications in 40 patients were analyzed. Then, three imaging methods were used to diagnose the features. Sensitivity and specificity were used to evaluate the diagnostic performance of three imaging methods for imaging features. Compared with professional doctors and biomarker algorithms, the sensitivity of CNN algorithm proposed was 90.6%, and DSC was 84.1%. Compared with traditional methods, the CNN algorithm has higher image resolution and wider and more accurate lesion area recognition and division. The three manifestations of soft tissue abscess, periosteum swelling, and bone damage were postoperative imaging features of bone and joint infections. In addition, compared with X-ray, CT examination and MRI examination were better for the examination of imaging characteristics. CT and MRI had higher sensitivity and specificity than X-ray. The experimental results show that CNN algorithm can effectively identify and divide pathological images and assist doctors to diagnose the images more efficiently in clinic.

## 1. Introduction

Bone and joint infection is not only a single bone and joint infectious disease, but also bone and joint infection is osteoarthritis caused by pathogenic microorganisms such as bacteria or viruses invading bone tissue and bone joint cavity. The biological cause of bone and joint infections is the invasion of pathogenic bacteria. According to the types of different pathogenic bacteria, bone and joint infections are classified into specific infection and non-specific infection; specific infection such as *Mycobacterium tuberculosis* causes bone and joint inflammation, and non-specific infection causes suppurative arthritis and bone marrow inflammation [1]. Clinically, bone and joint infections are often classified into acute infectious arthritis and chronic osteoarthritis. In addition, bone and joint infections include infections caused by trauma during surgery and implants. Suppurative bone and joint infections are classified into blood-borne and exogenous, and their pathogenic bacteria are mainly *Staphylococcus aureus*. Secondly, there are a small number of streptococci, *Staphylococcus haemolyticus*, *Brucella*, and *Escherichia coli* [2]. The common bone and joint infections in clinical orthopedics are suppurative bone and joint infections and osteomyelitis. There are roughly three stages in the course of suppurative bone and joint infections. The first stage is the inflammatory infiltration stage, in which inflammatory substances are gradually distributed widely in the bone marrow and a small amount of purulent fluid is visible. This stage usually occurs within three days after the onset of the disease. The second stage is the abscess stage, in which the articular exudate will increase, the pus will become more and more cloudy, leukocytes will increase, and the dissolved solvent will damage the periosteum. This stage occurs four to five days after the onset. The final stage, which occurs at five to six days after onset, is a rapid progression of the disease. The periosteum is destroyed as a whole, and purulent fluid spreads everywhere, seriously causing sepsis and even bone necrosis [3]. There are no clear boundaries between these three stages, and they can influence each other's evolution. Suppurative osteomyelitis usually occurs as complications of open fracture, internal fixation of fracture, diabetic foot, joint prosthesis replacement, and contaminated fracture [4]. It occurs in the tibia and femur, most of which are boils and carbuncles or purulent exudates from other parts of the body that reach bone tissue through the blood system, causing inflammatory symptoms of bone joints or bone tissue. Acute osteomyelitis usually onset is more urgent, with rapid progress, and patients can have high fever, local body swelling, swelling, tenderness, and other clinical symptoms. The clinical symptoms of chronic osteomyelitis are usually not obvious, so early diagnosis is difficult [5].

The article "Imaging Manifestations and Evaluation of Postoperative Complications of Bone and Joint Infections under Deep Learning" was retracted in 2023. Reasons: signs of a paper mill; compromised peer review; unreliable results or conclusions.

In recent years, with the rapid development of computer networks, deep learning has been gradually used in the medical field [6]. Deep learning is a part of machine learning and is one of the important methods to realize artificial intelligence. The process of deep learning in medical image analysis roughly first inputs the original image data and then preprocesses the image and reduces noise through the computer. Finally, a series of data information is obtained, and the purpose information is obtained through in-depth analysis of the obtained data information [7]. Deep learning mainly includes convolutional neural networks (CNNs), deep belief networks (DBNs), and stacked autoencoders (SAEs) [8]. CNN is an important algorithm application in deep learning, which was proposed in the 1960s. Compared with other algorithms, the biggest advantage is that there is a convolutional layer, and the convolutional layer can directly perform convolution operations on two-dimensional data without preprocessing, reducing the amount of parameter processing. Studies reported that CNN can not only predict the related diseases of the fracture site but also predict the various variable parameters of the patient during the examination based on the characteristics of the imaging elements [9]. The CNN model can improve the prediction accuracy of the fracture site by using the image features extracted by CNN and combining them with the multimodal model. Compared with independent image features, it has higher performance. There were also studies that set the training set to 40 sample data and the test machine to 10 sample data. CNN algorithm was employed to segment the CT image, and the similarity coefficient can reach 96.66% [10].

Therefore, this study intended to conduct imaging examination on patients with common postoperative complications of bone and joint infections through retrospective analysis to summarize their imaging characteristics. Moreover, deep learning algorithm was used to evaluate their imaging, so as to provide reference for better assisting doctors and utilizing the advantages of image-assisted diagnosis.

## 2. Methods

### 2.1. Imaging Techniques for Bone and Joint Infections

Chronic osteomyelitis, periosteal reaction, osteoporosis, bleeding, soft tissue abscess, and other complications usually occur after bone and joint infections. At present, the diagnosis of bone and joint infections mainly depends on clinical manifestations and imaging examinations. Since the clinical symptoms of complications lag behind the imaging manifestations, imaging examination is often used in treatment to improve the diagnostic accuracy of complications [11]. There are a variety of commonly used imaging methods, including X-ray examination, computed tomography (CT), and magnetic resonance imaging (MRI).

X-ray scan is the most basic imaging examination and evaluation method for bone and joint infections. When X-rays are taken, the scope should be expanded to cover all areas of the surgery and the area where the prosthetic material is implanted. X-rays, although not very clear, can show the general condition of bone and joint infections, osteolysis, soft tissue conditions, and other conditions at the surgical site. It can also show where the implant is and whether it has broken, fallen off, or loosened. However, X-ray films cannot show corresponding changes in complicated surgical anatomical areas, non-metallic implant materials, and related soft tissue changes after surgery, and their application is greatly limited [12].

The article "Imaging Manifestations and Evaluation of Postoperative Complications of Bone and Joint Infections under Deep Learning" was retracted in 2023. Reasons: signs of a paper mill; compromised peer review; unreliable results or conclusions.

CT is one of the important auxiliary diagnostics means in medical imaging. It mainly uses X-ray beam, gamma beam, and ultrasound. Through a very sensitive metal specific detector, the two are combined to perform a series of tomography scans on specific thicknesses of the body. Its advantages include fast scanning (each scanning time can be controlled within 40 ms at most), clear influence obtained from scanning, and high quality [13]. The radiation of CT scan is greater than that of X-ray, so CT scan is especially not suitable for women during pregnancy and lactation [14]. Moreover, because CT has the highest sensitivity to soft tissue, it can help detect bone and joint infections in orthopedic joints. The scanned data images are then uploaded to an electronic computer, which processes the received data images. Finally, multiplanar or reconstructed images were obtained, showing joints, damaged bone, soft tissue damage, periosteum reaction, and so on [15].

Compared to X-rays, soft tissue damage can be shown, but the images are not as clear as MRI images. MRI imaging technology was born around 1980. MRI imaging technology is often used for the auxiliary imaging diagnosis of soft tissue lesions, as well as the inspection of cartilage, bone tumors, and minor fractures [16]. MRI imaging technology in orthopedics uses the principle of magnetic resonance to receive electromagnetic signals of specific frequencies from the patient's body to generate MR signals. The electronic computer generates MR signals through spatial coding and image processing. Finally, multiangle sectional images of patients are obtained (transverse sectional images, coronal images, and sagittal images are commonly used) [17]. Compared with X-ray films, MRI images are multidirectional and three-dimensional and have high resolution, which are used for soft tissue examination. For CT scans, MRI does not cause radiation to the patient and can provide richer image information for the lesion. However, MRI is not as sensitive as X-rays and CT scans in the lungs. In addition, the examination time of MRI is longer than that of X-ray and CT scan, which requires long-term cooperation of patients and requires high compliance of patients [18].

The article "Imaging Manifestations and Evaluation of Postoperative Complications of Bone and Joint Infections under Deep Learning" was retracted in 2023. Reasons: signs of a paper mill; compromised peer review; unreliable results or conclusions.

These three methods are used to assist the diagnostic examination of bone and joint infections, but only by fully mining the image information can the auxiliary diagnostic function be played to the maximum extent.

### 2.2. Research Subjects

In this study, a total of 40 patients with postoperative bone and joint infections in the inpatient ward of the Department of Orthopedics of Orthopedics Hospital of Henan Province of Luoyang City were selected as the research objects. There were 27 male patients and 13 female patients. Their ages ranged from 35–89, with a mean age of 62 years. There were 32 patients with local pain, 10 with elevated body temperature, and 5 with local redness and swelling. With a history of between 3 and 12 months, 22 patients had a fracture and 18 did not.

Inclusion criteria were as follows: (i) patients aged between 35 and 89; (ii) patient's condition was clearly diagnosed as bone and joint infection disease according to the Treatment Guidelines for Orthopedic Diseases; (iii) all clinical information of patients was complete; (iv) all patients were willing to receive X-ray, CT, and MRI examinations; and (v) patients who had no typical clinical symptoms.

Exclusion criteria were as follows: (i) patients with age inconsistency; (ii) patients with other orthopedic complications; (iii) patients who were allergic to contrast agent and disinfection alcohol; and (iv) patients with mental problems or consciousness disorders.

All patients and their families in this study had signed informed consent, and the study had been approved by the Medical Ethics Committee of the hospital.

### 2.3. CNN Algorithm

The most classic algorithm in deep learning algorithms is the CNN algorithm. The CNN algorithm is used to deal with grid-like data and regression problems, including original imaging images and training data such as time series. The most basic structure is the LeNet-5 structure. The special linear operation method of CNN includes several important modules of input layer, convolution layer, pooling layer, and fully connected layer. The principle of CNN is that the input raw data will enter the fully connected layer after multiple layers or specific convolution operations and pooling operations. The data passing through the fully connected layer will pass through the mapping layer and become a fixed feature vector to form the calculation layer to reduce the parameter setting [18]. For each input data, a corresponding image information description will be obtained. The basic source structure of CNN is shown in Figure 1.

So far, all typical CNNs are composed of basic convolution operations. In general, the convolution operation is based on simple mathematical operations between two functions. Convolution operations have continuous and discrete types. In actual clinical practice, discrete convolution operations are more commonly used. The specific calculation method is as follows.

The article "Imaging Manifestations and Evaluation of Postoperative Complications of Bone and Joint Infections under Deep Learning" was retracted in 2023. Reasons: signs of a paper mill; compromised peer review; unreliable results or conclusions.

The convolution of continuity is defined as the following equation:

(1) $$\begin{array}{c} W\left(t\right)=\int_{-\infty }^{\infty }y\left(x\right)s\left(t-x\right)dx. \end{array}$$

Discrete convolution is defined as the following equation:

(2) $$\begin{array}{c} W\left(t\right)=\sum_{x=-\infty }^{\infty }y\left(x\right)s\left(t-x\right), \end{array}$$

in which *W*(*t*) represents the output result obtained, *y*(*x*) represents the input data, and *s*(*x*) represents the convolution kernel.

The convolution operation is summarized in two steps. First, it performs a linear operation on the input data. Then, according to the characteristics of each convolution kernel matrix, the sum of the elements at each position is multiplied to realize the entire convolution operation process, as illustrated in Figure 2.

The data information obtained by the convolution operation divides the input image data into fixed regions of interest through the pooling layer, and these regions of interest are used for feature expression. The most commonly used pooling method is maximum pooling, that is, it is expressed by calculating the maximum value of all the elements in a specific area, as shown in Figure 3.

### 2.4. Imaging Examination Process

All 40 patients received X-ray examination, CT examination, and MRI examination in sequence. The equipment used for X-ray was the Philips DR digital X-ray system of the Netherlands. Secondly, CT examination was performed on the patient. The equipment used for the CT examination was the GE whole-body spiral CT machine produced in the United States. The scanning voltage was 120 kV, the current was 300 mA, and the layer distance and layer thickness were both set to 0.5 mm. Then, enhanced continuous scanning was performed, the contrast agent was Uvisin, and the dose was 50 mL. Finally, the MRI examination was performed. The equipment used for the MRI examination was the US GE 1.5 T superconducting whole-body magnetic resonance scanner. The layer spacing and layer thickness were both set to 1 mm, and the reinforcing agent was gadopentetate meglumine. The dose was 0.1 mmol/kg. According to the spin echo method, perform T1WI (TR/TE500/20 ms) and T2WI (TR/TE4000/117 ms) scans The coronal layer, the sagittal layer, and the cross section were imaged separately, and the patient was scanned 30 seconds after the injection of the enhancer.

### 2.5. Evaluation Indexes of Imaging Manifestations of Postoperative Complications

The three complications of soft tissue swelling, bone damage, and periosteum reaction of patients were taken as imaging indicators by three imaging examination methods. Sensitivity and specificity were used to evaluate the imaging characteristics of complications.

The article "Imaging Manifestations and Evaluation of Postoperative Complications of Bone and Joint Infections under Deep Learning" was retracted in 2023. Reasons: signs of a paper mill; compromised peer review; unreliable results or conclusions.

### 2.6. Radiological Evaluation of Postoperative Complications of Bone and Joint Infections Based on CNN

To detect the performance of CNN applied in imaging technology, sensitivity and Dice similarity coefficient (DSC) were used for evaluation in this study. Biomarker algorithm was used to compare with CNN algorithm [19]. Sensitivity refers to the recognition performance of the image obtained by the algorithm compared with the original image to the lesion area. DSC represents the degree of overlap between the original image and the image processed by the algorithm. The larger the value of these two indicators was, the more accurate the result of the image was recognized and divided. The calculations were as follows:

(3) $$\begin{array}{c} \mathrm{sensitivity}=\frac{\left|M\cap N\right|}{\left|M\right|},\\ \mathrm{DSC}=\frac{2\left|M\cap N\right|}{\left|M\right|+\left|N\right|}, \end{array}$$

in which *M* represents the result of the clinician's identification and division of lesions, while *N* indicates that the algorithm recognizes and divides the results of lesions.

## 3. Results

### 3.1. The Processing Results of Images Based on CNN

Three imaging examination methods were used to identify and divide the imaging images of 40 patients with different degrees of postoperative complications of bone and joint infections, as presented in Figure 4. The images on the far left were all processed by using biomarker algorithm, the images in the middle were all identified and divided by imaging doctors, and the images on the far right were identified and divided by CNN algorithm. The resolution of the rightmost image was higher than that of the left image and the middle image, and the identification and division of the lesion area were broader and more accurate than those of the left image and the middle image, and the lesion area was clearer. In particular, the identification and division of MRI examination method were more accurate and intuitive compared with X-ray examination and CT examination. Therefore, the CNN algorithm had good application value for the recognition and division of imaging images. The lesion areas were marked in green.

### 3.2. Three Kinds of Imaging Processing Image Result Analysis

To quantitatively evaluate the CNN algorithm used in this research, sensitivity and DSC were used to evaluate the results of various identification and segmentation methods for pathological sites. The results are shown in Table 1. The image sensitivity evaluated by professional imaging doctors was 89.8%, and the DSC was 83.8%. The sensitivity of CNN algorithm was 90.6%, and the DSC was 84.1%. The sensitivity of biomarker algorithm was 83.1%, and the DSC was 84.7%. The recognition result of the CNN algorithm is basically the same as the result of the professional doctor's recognition and division of the lesion in the image and both of these two algorithms had higher sensitivity and DSC results than the biomarker algorithm. Therefore, the CNN algorithm used in this article can be applied to the recognition and classification of clinical diagnostic images.

The article "Imaging Manifestations and Evaluation of Postoperative Complications of Bone and Joint Infections under Deep Learning" was retracted in 2023. Reasons: signs of a paper mill; compromised peer review; unreliable results or conclusions.

### 3.3. Imaging Characteristics of Postoperative Complications by Three Imaging Examinations

Imaging analysis of 40 patients showed that postoperative complications of bone and joint infections mainly included soft tissue abscess, periosteum swelling, and bone damage. For soft tissue abscess, X-ray examination of 40 patients found that 29 patients had soft tissue abscess of varying degrees, subcutaneous tissue and muscle layer were reticulated, abscess site boundary was unclear, and thickness increased. CT scan showed that 34 patients had soft tissue abscess, and the patients' bone marrow was filled with purulent exudate with high density. MRI showed that 37 patients had characteristics of soft tissue abscesses, with low or ground intensity on T1W1-weighted images and high intensity on T2W1-weighted images and STIR sequences. Compared with the previous two methods, MRI showed a larger area of abscess and slight enhancement around the soft tissue where the abscess was present. For periosteal swelling, 30 patients had periosteal swelling reaction on X-ray examination, and the periosteal thickness was increased, and it was in the shape of strip and lace, and a small part was in the vertical shape. On CT scan, 33 patients showed slight periosteal swelling, which showed parallel strip and thickened bone. MRI did not detect significant periosteum swelling, which was suspected to be not significantly related to the differentiation of bone cortex distributed around the bone. For bone destruction, X-ray examination of the 40 patients revealed bone destruction in 23 of them, with osteoporosis in the epiphysis and slight thickening of the peripheral bone cortex. CT scan revealed bone destruction and obvious thickening of bone cortex in 30 patients. MRI examination revealed that 38 patients had hyperplasia and sclerosis of bone, with blurred epiphyseal boundary and multiple irregular patchy areas of bone destruction.  Table 2 and Figure 5 illustrate the details.

The article "Imaging Manifestations and Evaluation of Postoperative Complications of Bone and Joint Infections under Deep Learning" was retracted in 2023. Reasons: signs of a paper mill; compromised peer review; unreliable results or conclusions.

### 3.4. Evaluation Results of Imaging Characteristics of Different Inspection Methods

Three imaging methods were used to evaluate the sensitivity and specific indicators of the three imaging features of soft tissue abscess, periosteal swelling, and bone damage. As a result, it was found that the sensitivity and specificity of MRI examinations in particular were higher than those of X-ray examinations and CT scans, as shown in Figure 6.

## 4. Discussion

Bone joint infection refers to the infection of bone tissue and bone joint structure by bacteria and other pathogenic microorganisms (mainly *Staphylococcus aureus*). It releases toxic substances inside it, damaging normal bone tissue and joints and triggering an inflammatory response in the bone tissue or joints. Bone and joint infections can have multiple complications, including local swelling, pain, and bleeding. Bone joint infection included suppurative arthritis, *M*. *tuberculosis* bacillus infection, and osteomyelitis. It is caused by a highly erosive and fluid effusion of pus after infection. High pressure in the bone joint involves the normal bone tissue blood system and then destroys the normal bone tissue and bone structure [20]. If there is no timely intervention treatment, it will lead to bone and joint stiffness, joint cavity narrowing, and serious bone and joint deformity, affecting the normal life of patients. There are usually two ways to treat bone and joint infections. One is adopting antibiotics alone. However, if antibiotics are only given, patients should take them for a long time, resulting in drug resistance. Moreover, once microbial biofilms are formed on the surface of infected bone tissue, effective drug concentration is difficult to reach, and antibiotics will also lose efficacy [21]. Another method is debridement. Debridement first excises necrotic tissue, inactivated bone tissue, hematoma site, purulent exudate, and other parts by opening the bone and joint. Massive physiological saline and medical hydrogen peroxide should be used to wash the debridement site for many times and repeatedly to completely remove the infected site. After surgery, vancomycin and other corresponding antibiotics are combined therapy. However, if debridement is not complete or the debridement effect is not good, postoperative complications will cause secondary injuries to patients [22].

Clinically, bone and joint infections and their postoperative complications are generally diagnosed through clinical characterization, imaging, detection of biomolecular indicators, and laboratory examination of pathogenic microorganisms. However, postoperative complications of bone and joint infections have no typical characteristics in clinical manifestations. Most of them are local bone and joint pain, swelling, weakness, immobility of limbs, elevated body temperature, and so on. It is easily confused with osteomyelitis and other diseases. Therefore, imaging examination is often used as an auxiliary examination to identify. It was reported that in the diagnosis of lumbar intervertebral disc lesions, bone changes in the lumbar cone, lumbar facet joints, and other parts can be clearly shown in X-ray images. However, soft tissue lesions such as intervertebral discs and ligaments surrounding the spine are not visible. CT scans can show changes in bone as well as soft tissue structures that X-rays do not show. In addition, it can clearly indicate whether there is hematoma at the lesion site, whether there is periosteum reaction, the degree of influence on nerves, and so on [23]. Compared with CT scan, MRI can form three-dimensional reconstruction of bone tissue and joints, infection sites, microscopic bone diseases, and deep fractures through multiplane examination without the risk of radiation. In this study, three imaging examinations showed that soft tissue abscess, periosteum swelling, and bone destruction could be imaging features, and CT and MRI had better performance than X-ray examination.

The article "Imaging Manifestations and Evaluation of Postoperative Complications of Bone and Joint Infections under Deep Learning" was retracted in 2023. Reasons: signs of a paper mill; compromised peer review; unreliable results or conclusions.

Deep learning is an important component of machine learning. Many kinds of medical image data information are input by computer, and a series of intelligent algorithms are successively used to preprocess medical images, identify regions of interest, divide feature regions, extract feature regions, and carry out corresponding matching for feature regions [24, 25]. CNN algorithm is more classical. At present, CNN algorithm has been used to assist doctors in the diagnosis of various types of cancer detection, ophthalmic disease screening, osteoarthritis, and fracture diagnosis. It was found that using deep learning to reconstruct anteroposterior-lateral spinal images can simplify the complex features of 3D spinal models, and it can make sure that the features left behind are completely representative of the essential features of the whole model. It was also found that some typical characteristics of adolescent thoracolumbar malformation and the overall condition of thoracolumbar body could only be obtained through deep learning. This study also found that, compared with manual rendering and other algorithms, CNN algorithm had higher image quality, with 90.6% sensitivity and 84.1% DSC, which were both higher than those of the other two methods. It was suggested that CNN algorithm can be used as an auxiliary method for clinicians to deal with lesions.

The article "Imaging Manifestations and Evaluation of Postoperative Complications of Bone and Joint Infections under Deep Learning" was retracted in 2023. Reasons: signs of a paper mill; compromised peer review; unreliable results or conclusions.

## 5. Conclusion

In this research, CNN algorithm was used to process X-ray, CT, and MRI images of postoperative complications of bone and joint infections. It was found that CNN algorithm can effectively identify and classify pathological images, which can assist doctors to diagnose the images more efficiently in clinic. Soft tissue abscess, periosteum swelling, and bone damage can be used as imaging features of postoperative complications of bone and joint infections. In addition, imaging can well evaluate the postoperative complications of bone and joint infections and further guide doctors to make appropriate plans.

## Figures and Tables

**Figure 1:** Structure diagram of CNN's basic principle.

**Figure 2:** The convolution process of CNN.

**Figure 3:** Principle of maximum pooling operation.

**Figure 4:** Image processing results of three imaging methods. (a–c) X-ray examination images. (d–f) CT examination images. (g–i) MRI images. The leftmost images were the images processed by biomarker algorithm, the middle images were the results processed by doctors, and the rightmost images were the results processed by CNN algorithm.

**Figure 5:** The examination results of the imaging characteristics of postoperative complications in the three examination methods.

**Figure 6:** Evaluation indicators of the three inspection methods. (a) Sensitivity of the three inspection methods. (b) Specificity of the three inspection methods.

**Table 1:** Recognition and division results of images by three methods.

Method	CNN	Dr	Biomarker algorithm
Sensitivity (%)	0.906	0.898	0.831
DSC (%)	0.841	0.838	0.847

**Table 2:** Imaging diagnosis results of postoperative complications by different examination methods.

Method classification	X-ray	CT	MRI
Soft tissue abscess	29	34	37
Periosteum swelling	30	33	0
Bone destruction	23	30	38

## Data Availability

The simulation experiment data used to support the findings of this study are available from the corresponding author upon request.
